# GAP-43 Induces the Differentiation of Bone Marrow-Derived Mesenchymal Stem Cells into Retinal Ganglial-Like Cells

This article has been retracted.

**DOI:** 10.1155/2022/4949206

**Published:** 2022-04-21

**Authors:** Xiaoke Wang, Chi Ma, Lili Nie

**Affiliations:** ^1^Department of Neurosurgery, The Second Hospital of Jilin University, Changchun, 130000 Jilin, China; ^2^Department of Neurosurgery, The First Hospital of Jilin University, Changchun, 130021 Jilin, China; ^3^Department of Ophthalmology, The Second Hospital of Jilin University, Changchun, 130000 Jilin, China

## Abstract

Optic neuritis (ON) is a common neurological disease, and the transplant of retinal ganglion cells (RGCs) has been thought as a promising strategy for improving the injury of the optic nerve system. Bone mesenchymal stem cells (BMSCs) have the potential to differentiate into neural cells. Several studies have indicated that GAP-43 is related with the regeneration of nerve cells, while the effect of GAP-43 on inducing BMSC differentiation remains unclear. In this study, the BMSCs were separated from the rats and identified with flow cytometry assay. The GAP-43 expressed vectors were transfected into the BMSCs, and the biomarkers of RGCs such as PAX6, LHX2, and ATOH7 were used to observe by qRT-PCR. Moreover, the effect of GAP-43-induced BMSCs (G-BMSCs) on ON improvement was also verified with rat models, and the activity of MAPK pathway was measured with western blot. Here, it was found that GAP-43 could obviously promote the differentiation of BMSCs, and increased PAX6, LHX2, ATOH7, BRN3A, and BRN3B were observed in the process of cell differentiation. Moreover, it was also found that G-BMSCs significantly increased the abundances of NFL and NFM in G-BMSCs, and GAP-43 could also enhance the activity of MAPK pathways in BMSCs. Therefore, this study suggested that GAP-43 could induce the differentiation of bone marrow-derived mesenchymal stem cells into retinal ganglial cells.

## 1. Introduction

Optic neuritis (ON) is a neurological disease characterized with acute or subacute visual degeneration company with center visual impairment [1, 2]. The pathogenesis of the ON is complex, which could be contributed as infection, nonspecific inflammation, and demyelination, and thus, ON has been became as one of the most complex diseases in the field of ophthalmology [3], at present, hormonal treatment, immunosuppressor intervention, drug regulation, and plasma exchange. However, the side effects of those methods obtained in clinical observations have limited the application of those methods in the ON treatment. The strategy of RGC regeneration to reduce the injury of nerve cells could effectively improve the ON of the patients [4]. Recently, the therapeutic strategies involving the stem cells have been focused by increased researchers.

The stem cells such as mesenchymal stem cells (BMSCs) can differentiate as nerve cells, epithelial cells, and a variety of tissue cells [5]. BMSC is a type of adult stem cells came from the multiple tissues and has high potential to differentiate into multiple cells. The low immunogenicity of BMSCs could effectively reduce the inflammation and immunologic rejection of the body after transplant. Moreover, the accessibility and immunoregulatory capabilities promote BMSC treatment becoming a promising strategy for ON treatment [6, 7]. The recent studies have indicated that the level of GAP-43 may be connected with the nerve differentiation and growth [8]. GAP-43 locates on the membranes of nerve cells, and the expression of GAP-43 is related with the extension of axons [9]. Increased GAP-43 has also been found in the periods of neurite outgrowth during development of peripheral nervous systems [10, 11]. Thus, GAP-43 has been selected as a biomarker for axonal regeneration. However, whether GAP-43 upregulation could induce the differentiation of BMSCs into RGCs remains unknown.

This study attempted to investigate the effect of GAP-43 on BMSCs and explore whether the BMSCs could exhibit the similar biological characteristics of optical nerve cells after transfecting with GAP-43.

## 2. Material and Methods

### 2.1. Isolation and Culture of Rat BMSCs

The cells were isolated from the umbilical cords. In short, the umbilical cords were washed with 70% ethanol for three times, and the tissues of the vessels and amnion were removed. After that, the umbilical cords were cut up and then digested with collagenase II (270 U/mL) in an incubator with 37°C and 5% CO_2_ for 3 hours. Subsequently, Dulbecco's Modified Eagle Medium (DMEM)/F12 containing with 10% fetal calf serum (FCS), 100 U/ml penicillin, and 100 *μ*g/ml streptomycin was added into the cells for ending the digestion, and the liquid supernatant was removed after the centrifugation at 1000 rpm/min for 4 min. The cells were cultured with DMEM containing 10% FCS in an incubator with 37°C and 5% CO_2_, and the cells' subculture was performed when cell confluence was at 90%. Besides, the cell with CD45 negative and CD29 and CD90 positive were isolated for subsequent study.

### 2.2. Cell Transfection and Differentiation

3 × 10^3^ cells were seeded into T-25 culture flask, The cell transfection was performed when the confluence of cells was at 70%. In brief, 4 *μ*g of GAP-43 expressed vectors and Lipofectamine 2000 were, respectively, diluted and incubated with 250 *μ*l serum-free medium for 5 min, and then, the diluted vectors were mixed with diluted Lipofectamine 2000, and the configuration ratio was 1 : 1. After that, the mixture was incubated at 25°C for 20 min. Finally, 500 *μ*l of the mixtures was added into each well, and then, the cells were cultured for 24 hours. For cell differentiation, the BMSCs were transfected with GAP-43 expressed vectors and then cultured with DMEM. The morphology of the differentiated cells was observed every day.

### 2.3. Quantitative Real-Time PCR (qRT-PCR)

Total RNAs of the cells were extracted with TRIzol reagent according the manufacturer's instructions of the kit, and the concentration of the total RNAs was measured with ultraviolet spectrophotometry. After that, total RNAs were reversely transfected as cDNAs by reverse transcription kit. The PCR was performed according to the following cycling program: 95°C × 3 minutes for 1 cycle; 95°C × 20 seconds, 66°C × 10 seconds per cycle, and then -3°C per cycle for 4 cycles; and followed by 95°C × 10 seconds, 55°C × 15 seconds, and 70°C × 1 second for 40 cycles. U6 was used as a reference control, and the relative expression levels were calculated with 2^−*ΔΔ*Ct^ method.

### 2.4. Western Blot

Total proteins of the cells were extracted with RIPA buffer on the ice, and BCA kit purchased from Thermo Fisher Scientific (New York, USA) was used to detect the concentration of the extracts. After that, 30 *μ*mL of the extracts was separated with sodium dodecyl sulfate-polyacrylamide gel electrophoresis (SDS-PAGE), and then, proteins were transferred on the polyvinylidene fluoride (PVDF) membranes by wet-transfer method. After that, the membranes were blocked with 5% fat-free milk for 2 hours and then were incubated with the related first antibodies overnight at 4°C (all antibodies were purchased from Abcam, UK). Subsequently, the membranes were washed with TBST for three times (15 min/time), and then, the membranes were incubated with the second antibodies for 2 hours at room temperature. Finally, the expression of the proteins was observed with a chemiluminescence system.

### 2.5. Axonal Outgrowth Assay

For the measurement of axonal outgrowth, the G-BMSCs were cultured in 6-well plates. 4% paraformaldehyde (PFA) was added for cell fixation for 20 min, and then, cells were strained with anti-*β*-III-tubulin (Ab52623, AmyJet Scientific Inc, Wuhan, China) at 4°C overnight. After that, the cells were further incubated with Alexa Fluor 647-tagged antibody (1 : 500; Life Technologies, USA) at 25°C for 2 hours. GFP^+^ and DAPI^+^ RGCs were imaged on a Zeiss Axio Observer inverted microscope using a 10x objective to measure neurite outgrowth.

### 2.6. Flow Cytometry

The surface biomarkers of BMSCs were analyzed by flow cytometry, and the antibodies conjuncted with fluorescein isothiocyanate were used to observe the expressions of CD29, CD90, and CD45 in the cells.

### 2.7. Statistical Analysis

The experiments in this study were performed for three times, independently. The results were analyzed with the SPSS software and were exhibited with Graph Prism 8.0. Moreover, Chi-squared test or ANOVA with Tukey's post hoc test was used to calculate the difference of two groups, and *P* < 0.05 meant that the difference of the data is statistically significant.

## 3. Results

### 3.1. Characterization of BMSCs

To keep the quality of the cells, the phenotype of the isolated cells was observed under the microscope. The result showed the cells with round shape at the initial stage of culture exhibited triangular, fusiform, or spindle shapes after culture for 48 hours. After 6-8 days, most of subculture cells exhibited spindle shapes. After culture for 100 days, the cells did not show the sign of senescence or differentiation (Figure 1(a), *P* < 0.01). Moreover, the results of immunofluorescence staining showed that BMSC expressed antigens of CD29 and CD90 (Figure 1(b), *P* < 0.01). Moreover, no expression of the CD45, the biomarker of hematopoietic cells, was observed (Figure 1(b), *P* < 0.01). Hence, these findings suggested that purified BMSCs have been isolated successfully.

### 3.2. GAP-43 Promoted the RGC-Like Cell Differentiation of BMSCs

To identify the characters of the differentiated BMSCs, the cells were selected and identified by flow cytometry assay, and the expression of the specific biomarkers in RGCs was also observed by qRT-PCR. At day 6, it was found that the expression levels of PAX6, LHX2, and ATOH7 significantly increased compared with the undifferentiated BMSCs (Figures 2(a)–2(c), *P* < 0.01). By day 8, increased BRN3A and BRN3B were also observed in the BMSCs transfected with GAP-43 expressed vectors (Figures 2(d) and 2(e), *P* < 0.01). Therefore, these observations suggested that the GAP-43-induced BMSCs exhibited RGC-like characters.

### 3.3. G-BMSCs Developed Neurite Networks and Exhibited Characters of RGCs In Vitro

To confirm whether G-BMSCs could effectively promote the regeneration of axons, at day 22, the structure of the BMSCs was observed by axonal outgrowth assay, and the expression levels of axon-related proteins was measured by western blot. The results showed that G-BMSCs exhibited obvious axon generation compared with the undifferentiated BMSCs (Figure 3(a)). Moreover, the western blot showed that NFL and NFM were significantly upregulated in BMSCs transfected with GAP-43 expressed vectors compared with the BMSCs transfected with negative control after culturing for 22 days (Figures 3(b) and 3(c), *P* < 0.01).

### 3.4. MAPK Signaling Pathway Was Activated in the BMSCs Induced by GAP-43

To delve the mechanism of the GAP-43 on the difference of BMSC, the upregulated MAPK pathway was observed by western blot. The results showed compared with the BMSCs transfected with NC-vectors, the BMSC cells with upregulated GAP-43 exhibited high activity of the MAPK pathways, and the abundances of JNK, p-JNK, P38, p-38, ERK, and p-ERK were increased significantly (Figure 4, *P* < 0.01). Therefore, those observations suggested that GAP-43 could induce the differentiation of BMSCs into RGCs via activating MAPK pathway.

## 4. Discussion

The transplant of the RGCs has been identified as a promising strategy for the treatment of eye-related diseases [12]. BMSCs are characterized with pluripotent abilities to differentiate multiple types of the cells including nerve cells, which may be used for producing the RGC-like cells. Moreover, the low immunogenicity makes it possible that BMSC transplant could repair the impaired organ with only subtle immunological rejection [13]. Various studies have focused on the application of BMSCs in improving the injury of nerve system induced by inflammation and oxygen stress [14]. In this study, the related regulation mechanism of GAP-43-induced the differentiation of BMSCs to RGC-like cells was investigated to provide some reference for ON treatment.

BMSC transplant has been thought as a promising strategy for the treatment of some neural diseases, and the differentiation of the BMSCs to Schwann cells has been indicated by several studies. CD29 and CD90 have been confirmed as the special biomarkers of BMSCs, and they have been used for identification of BMSCs by multiple studies [15]. In this study, BMSCs were isolated from the organ of the rats, and the related biomarkers of BMSCs were identified, and the cells showed high expression of CD29 and CD90. Moreover, reduced CD45 was also observed in the cells. The study has indicated that GAP-43 was significantly upregulated in the differentiation of RGCs, and increased GAP-43 could promote the survival and regeneration of RGCs [16, 17]. In this study, it was found that the BMSCs transfected with GAP-43 exhibited RGC-like properties. Moreover, increased PAX6, LHX2, and ATOH7 were observed in the G-BMSCs at prophase of cell culture. PAX6, LHX2, and ATOH7 serve as important factors for the development of mammal retinas. Badea et al. have confirmed that ATOH7 mutation could induce the optic nerve hypoplasia [18]. Besides, upregulated BRN3A and BRN3B were also measured during the subsequent cell culture. BRN3A and BRN3B serve as critical roles in development of mammal optic system, and thus, they are confirmed as important biomarkers of RGCs [19, 20]. Therefore, these proofs suggest that the GAP-43 could induce the differentiation of BMSCs into RGC-like cells.

Neuroaxonal loss induced by demyelination and RGC injury is major reason leading the deterioration of ON, and the study has found that axon regeneration could effectively improve the symptom of the patients [3, 21]. Therefore, how to promote the regeneration of axons is a critical issue in the development of the therapeutic strategy for ON. In this study, obvious neuroaxonal generation was observed in the BMSCs transfected with GAP-43. Moreover, it was found that NFL and NFM were significantly upregulated during the cell culture of G-BMSCs. The deficiency of NFL is related with the progression of ON. Several studies have indicated that NFL and NFM are significantly downregulated in the eyes of the patients with ON, and the expression of NFL has always been selected as a biomarker for the diagnosis of optical system [22, 23]. These proofs suggest that GAP-43 could induce the differentiation of BMSCs into RGC-like cells.

The differentiation of BMSCs is related with the change in activation of multiple pathways, such as Wnt/*β*-catenin, MEK/RRK, and Notch. Zhang et al. have observed that the expression of *β*-catenin was significantly upregulated in the osteogenic cells differentiated by BMSCs [24]. Several studies have confirmed that inactivated MAPK pathway is observed in RGCs and axons after suffering injury [25]. In this study, activated MAPK pathway was observed in the BMSCs transfected with GAP-43. Inactivated MAPK pathway is related with the RCG apoptosis, and inhibition of MAPK pathway has been contributed as a direct mechanism of methylprednisolone-mediated degeneration and apoptosis of RGCs in ON rat models [26]. Moreover, the study has also indicated that 7,8-dihydroxyflavone could effectively improve the survival of RGCs via activating MAPK/ERK pathway [27]. Hence, this study suggested that GAP-43 plays an important role in the differentiation of BMSCs to RGC-like cells, and increased GAP-43 could activate MAPK pathway in G-BMSCs.

## Figures and Tables

**Figure 1:** BMSCs were isolated successfully. (a) The morphology of BMSCs was observed and imaged by light microscope (magnification, ×100). (b) The biomarkers of BMSCs were identified with flow cytometry assay.

**Figure 2:** GAP-43 promoted the RGC-like cell differentiation of BMSCs. (a–e) The relative expression levels of PAX6, LHX2, ATOH7, BRN3A, and BRN3B were measured with qRT-PCR (^∗∗^*P* < 0.01).

**Figure 3:** G-BMSCs developed neurite networks and exhibited characters of RGCs. (a) The neurite networks were observed by axonal outgrowth assay. (b, c) The mRNA levels of NFL and NFM (^∗∗^*P* < 0.01).

**Figure 4:** MAPK signaling pathway was activated in GAP-43-induced BMSCs. (a–g) The expression levels of JNK, p-JNK, P38, p-38, ERK, and p-ERK were measured by western blot (^∗∗^*P* < 0.01).

## Data Availability

Data to support the findings of this study is available on reasonable request from the corresponding author.
